This article has been retracted.

# A Pavement Crack Detection Method Based on Multiscale Attention and HFS

**DOI:** 10.1155/2022/1822585

**Published:** 2022-01-27

**Authors:** Chun Li, Yu Wen, Qingxuan Shi, Fang Yang, Hongyan Ma, Xuedong Tian

**Affiliations:** ^1^School of Cyber Security and Computer, Hebei University, Baoding 071002, China; ^2^Hebei Machine Vision Engineering Research Center, Hebei University, Baoding 071002, China; ^3^Institute of Intelligent Image and Document Information Processing, Hebei University, Baoding 071002, China; ^4^School of Mathematics and Information Science, Hebei University, Baoding 071002, China

## Abstract

To solve the problem of low detection accuracy due to the loss of detailed information when extracting pavement crack features in traditional U-shaped networks, a pavement crack detection method based on multiscale attention and hesitant fuzzy set (HFS) is proposed. First, the encoding-decoding structure is used to construct a pavement crack segmentation network, ResNeXt50 is used to extract features in the encoding stage, and a multiscale feature fusion module (MFF) is designed to obtain multiscale context information. Second, in the decoding stage, a high-efficiency dual attention module (EDA) is used to enhance the ability of capturing details of the cracks while suppressing background noise. Finally, the membership degree of the crack is calculated based on the advantages of the HFS in multiattribute decision-making to obtain the similarity of the crack, and the binary image after segmentation is judged by the hesitation fuzzy measure. The experiment was conducted on the public road crack dataset Crack500. In terms of segmentation performance, the evaluation indexes Intersection over Union (IoU), Precision, and Dice coefficients of the proposed network reached 55.56%, 74.26%, and 67.43%, respectively; in terms of classification performance, for transversal and longitudinal cracks, the classification accuracy was 84% ± 0.5%, while the block and the alligator were both 78% ± 0.5%. The experimental results prove that the crack details detected by the proposed method are more abundant, and the image detection effect of complex topological structures and small cracks are better.

## 1. Introduction

As the lifeblood of the national economy, the quality of pavement operation plays a vital role in the normal progress of production and life. Due to the pressure and climatic effects of heavy loads throughout the year, most of the roads have suffered from varying degrees of disease. Cracks are one of the common pavement diseases. If not discovered and treated in time, it will affect the service life of the road surface [1]. Traditional detection methods are inefficient and costly, and cracks show problems such as complex topology, poor continuity, low contrast, and strong noise [2], which brings challenges to the automatic detection of road cracks. Therefore, it is necessary to design an efficient automatic road crack detection method.

Based on the traditional image processing method, it is the initial attempt to automatically detect road cracks. Akagic et al. [3] proposed a crack image detection method based on the Otsu threshold and histogram. Although this method is efficient, the crack area can be accurately found only when the crack pixel is darker than the surrounding pixels. Medina et al. [4] used the wavelet transform method to detect cracks, which not only was susceptible to the contrast between crack pixels and surrounding pixels, but also could not detect cracks with poor continuity. To improve the effect of detecting continuous cracks, the minimum path selection method [5] is proposed to detect cracks from a global perspective, which effectively enhances the continuity of fractured cracks. Although the minimum path selection method performs crack detection from a global perspective, its detection performance is still unsatisfactory when dealing with cracks with disordered shapes or low contrast with surrounding pixels. It can be seen that automatic detection of road cracks is still a difficult task for researchers.

In recent years, deep learning has been applied to road crack detection tasks due to its outstanding feature extraction capabilities. Pauly et al. [6] cropped each crack image into a patch, and then the patch was classified as crack or noncrack after neural network training. Although this method was very efficient, it produced false detections. To further improve its detection accuracy, semantic segmentation algorithms based on the encoding-decoding architecture are widely used. Lau et al. [7] introduced U-Net to road crack detection. The network introduced skip connections into the encoding-decoding architecture, which helped to preserve rich image details, thereby improving the detection accuracy. Although U-Net performs well in the field of image segmentation, the crack area of the crack image is much smaller than the background area. Cao et al. [8] replaced the U-Net encoder with ResNet34 to deal with the loss of spatial information caused by continuous pooling. Effectively avoiding gradient disappearance or gradient explosion, Chen et al. [9] embedded a global context module in the U-Net network structure to give the network the ability to capture global context information, which is conducive to the detailed segmentation of pavement crack images. Augustauskas and Lipnickas [10] introduced a kind of attention based on the U-shaped network. The force gate model suppresses background noise and strengthens the ability of the network to capture detailed features of cracks. Fan et al. [11] proposed an end-to-end pixel-level road crack detection network. By building multiple expansion convolution modules to help the network obtain the multiscale context information of the cracks, a hierarchical feature learning module is designed to integrate low-level features and high-level features. The designed multiscale output feature map has better performance in fracture information inference, thereby improving the robustness and universality of the network. Ali et al. [12] implemented a deep fully convolutional neural network based on residual blocks. For the extreme imbalance between target and background pixels in crack images, a local weighting factor was proposed to effectively reduce the trouble caused by pixel imbalance to the network; a crack image dataset with different crack width directions and a location dataset were developed for researchers to use for training, validation, and testing. Fan et al. [13] proposed a road crack automatic detection and measurement network based on probability fusion. Through the designed integrated neural network model, satisfactory crack detection accuracy is obtained; according to the predicted crack map, the width and length of the crack can be measured effectively. Wang et al. [14] proposed a semisupervised semantic segmentation network for crack detection. The model extracts multiscale crack feature information through Efficient-UNet; it greatly reduces the workload of labeling while maintaining high labeling accuracy. Wang et al. [15] used a neural network to detect pavement cracks and applied a principal component analysis to classify the detected pavement cracks. The crack types were divided into transversal, longitudinal, cracked cracks. The accuracy scored higher than 90%. Nevertheless, patch classification is only suitable for rougher classification tasks. Cubero-Fernandez et al. [16] classified the discontinuous cracks in an image as a whole, though they did not consider the spatial distribution relationship between the cracks.

Existing road crack detection methods enhance the extraction and classification capabilities of crack features through global context modules, attention mechanisms, and principal component analysis methods to improve detection and classification accuracy. Because of the crack image detection, the foreground pixels are relatively small and have different lengths and widths. If a natural image detection method with a large proportion of foreground pixels is used, the effect is often poor, and eventually the information of the detected cracks will be lost, thereby affecting the detection effect. Therefore, this paper proposes a road crack detection method based on multiscale attention and HFS. The method is mainly divided into two tasks: semantic segmentation of the crack image [1] to realize the separation of the crack area and the noncrack area and the classification of the segmented binary image. For the first task, the proposed solution uses rectangular soft pooling instead of global average pooling, which effectively extracts long and narrow fracture feature information; rectangular pooling is used to fuse multiscale feature information to expand the receptive field of the network, so that the small proportion of crack information in the image is also noticed, thereby improving the accuracy of segmentation, using channel and spatial attention to assign the importance of two-dimensional weights, and based on this importance to improve the useful information for crack identification and suppress useless information. Different from existing segmentation methods, our proposed solution is more suitable for segmenting images with unbalanced aspect ratios such as cracks. For the second task, the core of the classification algorithm of the proposed solution is to define the number of crack branches, the number of inflection points, and the centroid distance index and use the multiattribute decision-making of HFS to calculate the similarity to classify. Compared with the existing classification algorithms, our method provides a more detailed qualitative classification method, which can derive the crack image category from the comprehensive analysis of multiple indicators.

The main contributions of this article are as follows:

1. Based on the encoding-decoding architecture, a multiscale feature fusion module is designed to obtain more receptive fields, so as to improve the network's ability to recognize disordered cracks.
2. Design an efficient dual attention module to realize the information interaction between spatial features and channel features, so as to improve the network's anti-interference ability and network feature extraction ability.
3. The segmented binary image is analyzed by the connected domain algorithm, and the advantages of hesitant fuzzy sets in multiattribute decision-making are used to calculate the fracture multiattribute membership degree to obtain the similarity of the fractures to determine the fracture category.

The rest of the paper is structured as follows: the second part elaborates the fracture segmentation network based on multiscale attention and the crack classification method based on hesitant fuzzy sets; the third part analyzes and discusses the experimental results; the fourth part summarizes the paper.

## 2. Materials and Methods

### 2.1. Fracture Segmentation Network Based on Multiscale Attention

The overall structure of our proposed solution Multiscale Attention Crack Segmentation Network (MACSNet) is shown in Figure 1.

The network consists of Encoders (E1, E2, E3, E4), Decoders (D1, D2, D3, D4), an EDA module and a MFF module. When designing the network structure, considering that the proportion of crack pixels in the image is small, the network structure should not be too deep, but a certain degree of accuracy must be ensured. Therefore, the encoder uses ResNeXt50 as the basic network to extract the characteristics of the input crack image. Its essence is grouped convolution, and the algorithm performance is improved by increasing the number of branches. The encoder in this structure retains the first five feature extraction modules of ResNeXt50, which are named pooling and E1-E4, respectively, as shown in Figure 1.

In addition, to obtain multiscale features, a multiscale feature fusion operation is performed after the E4 encoder to better extract the multiscale context information from the crack image and optimise the segmentation effect, as well as to incorporate efficient dual attention into the jump connection of encoding and decoding. The module allows the network to effectively integrate the low-level spatial resolution and the high-level semantic information, while further paying attention to the area where the crack is located. The module also combines the advantages of subpixel convolution and bilinear interpolation in the decoder D1–D4 and design a parallel feature fusion structure to sequentially restore image resolution and detailed information. To further integrate spatial resolution and high-level semantic information, inspired by dense connection [17], D3 and D4 are, respectively, upsampled twice. Then, the results of the 3 levels are superimposed in a concatenate manner.

#### 2.1.1. Efficient Dual Attention Module

The features extracted in the fracture segmentation network must not only contain enough spatial information to locate small-scale cracks, but also contain rich semantic information to effectively distinguish between cracks and other interference information. The Efficient Channel Attention (ECA) [18] strengthens the feature propagation ability of the channel dimension. Compared with the classic channel attention mechanism [19–21], it does not require dimensionality reduction operations to capture rich semantic information. However, in the high-level features of the cracks, it lacks sufficient spatial information. Inspired by the cascade of channel and spatial attention in Convolutional Block Attention Module (CBAM) [22], this paper introduces the importance of pooling in the ECA attention mechanism [23] to fuse channel weight information and spatial position information, while also designing an efficient dual attention module EDA. Its operating principle is shown in Figure 2, which can make the network better distinguish the importance of crack features and further improve the accuracy of the segmentation network.

The module is divided into upper and lower branches:

(1) The upper branch is used to capture channel attention features. This branch first obtains the global receptive field through a global average pooling operation and then uses 2D convolution to achieve channel interaction, taking each channel and its *K*=3 neighbouring channels to generate local cross-channel attention information, as shown in
  (1) $$\begin{array}{c} F_{i}=\sigma \left(\sum_{j=1}^{K}F_{j}\cdot Y_{i,j}\right),\;Y_{i,j}\in \Omega_{i,k}, \end{array}$$
 where *F*_*j*_ represents the one-dimensional convolution of size *K* , Ω_*i*,*k*_ represents the set of *K* adjacent channels of the input feature *Y*_*i*_, *σ* represents the sigmoid activation function, and *F*_*i*_ represents the attention information of *K* adjacent channels to the current channel.
(2) The next branch is used to capture spatial attention features, which trains a weight function on the original feature map, similar to the attention function, and then to perform a weighted average with the original image. Then, the weight function distributes the spatial feature weights through the sigmoid to obtain the importance space attention, as shown in
  (2) $$\begin{array}{c} F_{s}=\sigma \left(\text{conv}2\;d\left(\frac{\sum_{i\in R}a_{i}\cdot \;\exp\left(G\left(a_{i}\right)\right)}{\sum_{j=R}\exp\left(G\left(a_{j}\right)\right)}\right)\right), \end{array}$$

where *a*_*i*_ represents the original feature map, exp makes the weight value nonnegative and easy to optimise, and *G* represents the weight function after the network obtains *G* through training to enhance specific features.

#### 2.1.2. Multiscale Feature Fusion Module

ASPP [24] obtains multiscale fracture feature information through hole convolution with different sampling rates and has achieved good results in classification and segmentation tasks. Because the fracture shape is long and narrow, only the adaptive average pooling is not enough to obtain the global context information of the fracture, while the strip pooling [25] can obtain the long-distance dependence. Inspired by this, the Soft-Pool [26] of strip shape is introduced on the basis of ASPP, which effectively increases the global features. This research combines the advantages of ASPP and Soft-Pool to design a multiscale feature fusion module MFF, which effectively combines global information and multiscale context information, reducing the discontinuity problem in fracture segmentation, as shown in Figure 3.

The MFF first undergoes a 1 × 1 convolution to reduce the dimensionality and then obtains a multiscale parallel structure through a variety of sampling rates and pooling methods. The first three branches of the parallel structure fuse hole convolutions with different sampling rates to obtain multiscale information. The latter of the two branches obtains global information that is more suitable for the shape of the crack through soft pooling of the strip shape. Strip soft pooling mainly uses the maximum approximate *R* in the activation area. Each activation *a*_*i*_ with index *i* applies a weight *W*_*i*_, and the weight is equal to the natural number of activation values divided by the sum of the natural exponents of all activation values, as shown in the following equation:

(3) $$\begin{array}{c} W_{i}=\frac{e^{a_{i}}}{\sum_{j=R}e^{a_{j}}}. \end{array}$$

This weight is multiplied by the corresponding activation value to make a nonlinear transformation together, and the higher activation has a more obvious impact on the output. Since pooling is performed in a high-dimensional feature space, highlighting the maximum activation effect is more reasonable than directly selecting the maximum value. The output value of the Soft-Pool operation is obtained by summing all of the weighted activations in the kernel neighbourhood *R*, as shown in the following equation:

(4) $$\begin{array}{c} a=\sum_{i\in R}W_{i}*a_{i}, \end{array}$$

#### 2.1.3. Decoder Module

The decoder restores the image resolution through an upsampling method. A common upsampling method is bilinear interpolation, which restores the resolution through the neighbouring pixel values, but the restored boundary is blurry. The introduction of subpixel convolution in superresolution [27] can make the details of the image clearer. Therefore, the decoding block shown in Figure 4 is designed by combining bilinear interpolation and subpixel convolution. The upper branch undergoes general operations, such as a 1 × 1 convolution, batch normalisation, and ReLU, and then applies bilinear interpolation for upsampling; the lower branch is subpixel convolution. After the fusion of the two branch features, the detailed information of the detected cracks is more complete, and the amount of calculation added is small. The structure of the decoder module is shown in Figure 4.

### 2.2. Crack Classification Algorithm Based on Hesitant Fuzzy Sets

The type of crack is an important index to evaluate the quality of the pavement. The evaluation of different types of cracks directly affects the decision-making of different maintenance strategies. This section extracts the five features of the number of cracks in the image, the number of inflection points, the average centroid distance, the angle between centroids, and the area of the cracks while using the decision-making advantages of hesitation fuzzy set theory to realize crack classification.

On the basis of Zadeh fuzzy set theory [28], Torra proposed a hesitating fuzzy set [29], which allows the degree to which the element belongs to the set to be given in the form of a set of multiple possible values, in order to effectively characterize the uncertainty in decision-making. In the formula below, X is a nonempty set and call E the hesitant fuzzy set:

(5) $$\begin{array}{c} E=\left\{<x,h_{E}\left(x\right)>|x\in X\right\}, \end{array}$$

where *h*_*E*_(*x*) represents the set of membership degrees of the element *x* in the set *X* to the set *E*. It is a possible membership set in [0,1]; then, *h*=*h*_*E*_(*x*) is called the hesitant fuzzy element. *P* and *Q* are two hesitant fuzzy sets about *X*={*x*_1_, *x*_2_, *x*_3_,…, *x*_*n*_}; then the generalized hesitant fuzzy distance measure between them is shown in

(6) $$\begin{array}{c} d_{ghn}\left(P,Q\right)=\frac{1}{n}\sum_{i}^{n}{\left[\frac{1}{l_{x_{i}}}\overset{l_{x_{i}}}{\underset{j=1}{\sum }}{\left|h_{P}^{\sigma \left(j\right)}\left(x_{i}\right)-h_{Q}^{\sigma \left(j\right)}\left(x_{i}\right)\right|}^{\lambda }\right]}^{1/\lambda },\\ s\left(P,Q\right)=1-d_{ghn}\left(P,Q\right), \end{array}$$

where *n* is the number of elements in the set *X*, *h*_*P*_^*σ*(*j*)^(*x*_*i*_) and *h*_*Q*_^*σ*(*j*)^(*x*_*i*_) are the *j*-th largest values in *h*_*P*_(*x*_*i*_) and *h*_*Q*_(*x*_*i*_), respectively, *s*(*P*, *Q*) is the corresponding similarity, and *λ* is the control parameter. The generalized hesitant fuzzy distance measure gives the distance calculation formula of two hesitant fuzzy sets under multiple attributes and multiple indicators. The smaller the distance, the greater the similarity between them. This helps to realize the measurement of multiattribute similarity.

After detecting the pixel area containing the crack, the connected area algorithm is used to divide the crack into independent crack branch targets. After analysis, the number, area, centre position coordinates, and approximate length and the width of the crack branches are obtained. To further analyze the spatial distribution relationship between adjacent cracks, a Minimum Enclosing Rectangle (MER) [30] is generated for each crack branch target. As shown in Figure 5, each MER record includes the position coordinates of the crack branch target, height, and width. Then by calculating the MER information of the two branch targets, it is judged that C1 and C2 can be merged into a new branch target. When two types of crack branches appear in the crack image, the types are divided according to the pixel weight.

**Definition 1 .**

*C*_*q*_ represents the input road crack binary image and *C*_*q*_*j*__ represents any crack binary image in the dataset (*j*=1,2,…, *n*, *n* is the total number of road crack binary images in the dataset).

**Definition 2 .**

*N*_*P*_ is the hesitant fuzzy evaluation attribute of the crack image.

**Definition 3 .**

The cracks are divided into four types: transversal, longitudinal, block, and alligator, which are divided into T, V, M, and C.

#### 2.2.1. Hesitating Fuzzy Attribute Index

*(1) The Number of Branches IndexT*_num_. By analyzing the number of branch targets in the crack image, the degree of similarity between the two images *C*_*q*_*j*__ and *C*_*q*_ is evaluated. When the number of branches is greater than or equal to 3, the probability of being M or C type is greater. When the number of branches is less than 3, the probability of being T or V type is greater.

**Definition 4 .**

The membership function of the number of branches is

(7) $$\begin{array}{c} \mu_{T_{\text{num}}}\left(C_{q},C_{q_{j}}\right)=e^{\left(-\text{len}\left(C_{q}\right)/\left(\text{len}\left(C_{q_{j}}\right)\right.+\beta \right)}, \end{array}$$

where len(*C*_*q*_) is the number of crack branches in the input crack image, len(*C*_*qj*_) represents the number of crack branches in any image in the dataset, and *β* is the balance parameter.

*(2) Inflection Point IndexT*_ang_. To further divide the cracks into M, C type or T, V type, the Freeman code is introduced to reencode the crack image to obtain the boundary sequence of the crack and the number of substantial inflection points. When the number of inflection points is greater than or equal to 2, the probability of being M and C types is high.

**Definition 5 .**

The membership function of the inflection point index is

(8) $$\begin{array}{c} \mu_{T_{\text{ang}}}=\frac{1}{1+e^{T_{\text{ang}}\left(C_{q_{j}}\right)+\beta }}. \end{array}$$

*(3) Centroid Distance IndexT*_dis_. The centroid average distance (dis) of the crack branches in the image judges whether it is M type or C type. When dis is less than the threshold 0.5, it is C type, and when it is greater than or equal to 0.5, it is M type. Figure 5 shows the average distance between the judgement and the calculated centroids. When the average distance between the centroids of *C*_*q*_*j*__ and *C*_*q*_ is closer, the similarity is higher.

**Definition 6 .**

The membership function of the centroid distance index is

(9) $$\begin{array}{c} \mu_{T_{\text{dis}}}=\frac{1}{1+e^{T_{\text{dis}}\left(C_{q_{j}}\right)+\beta }}, \end{array}$$

where *T*_dis_(*C*_*q*_*j*__) is expressed as *T*_dis_(*C*_*q*_*j*__)=(*S*_*C*1_/(*S*_*C*1_+*S*_*C*2_+*S*_*C*3_))*∗*dis_1_+(*S*_*C*2_/(*S*_*C*1_+*S*_*C*2_+*S*_*C*3_))*∗*dis_2_; the centroid distance weight is larger when the crack area accounts for a larger proportion; *β* is the balance parameter.

*(4) Centroid Included Angle IndexT*_*flg*_. The angle between the diagonal of MER and the transversal direction judges whether it is T type or V type. The diagonal direction always faces the centre of the mass and the direction of the crack. When the included angle is 0°–45° or 135°–180°, the crack type is T; when the included angle is 45°–135°, the crack type is V, as shown in Figure 6.

**Definition 7 .**

The membership function of the centroid included angle index is

(10) $$\begin{array}{c} \mu_{T_{flg}}\left(C_{q},C_{q_{j}}\right)=\left\{\left({\text{Lev}}_{flg\_j},h_{S_{flg\_j}}\right)j=T,V\right\}, \end{array}$$

where Lev_*f*lg_*j*_ represents the type of angle between the diagonal of the MER and the transversal direction and *h*_*S*_flg_*j*__ represents the degree of membership corresponding to the angle.

*(5) Crack Area IndexT*_*s*_. According to the ratio of the crack area in the image to the original area, the importance of crack branches in the image is divided into three types: light (s), medium (m), and heavy (l). When there are multiple types of cracks in an image of a crack, the type of cracks in the image is judged according to the importance.

**Definition 8 .**

The membership function of the fracture area index is

(11) $$\begin{array}{c} \mu_{T_{S}}\left(C_{q_{j}}\right)=\left\{\left({\text{Type}}_{S\_j},h_{SS_{\text{type}\_j}}\right)|j=s,m,l\right\}, \end{array}$$

where Type_*S*_*j*_ represents the type of fracture importance and *h*_*SS*_*t*ype_*j*__ represents the degree of membership corresponding to different types.

The abovementioned indexes *T*_num_, *T*_dis_, and *T*_flg_ define the classification of pavement diseases according to the “China Highway Technical Condition Evaluation Standard,” and the indexes *T*_ang_ and *T*_*s*_ supplement the abovementioned indexes. *T*_num_ represents the number of branches in an image, used to determine whether it is a unidirectional crack or a network crack; *T*_dis_ represents the centroid distance between multiple branches in an image, which is used to further judge whether the network crack is an alligator or a block crack; *T*_*flg*_ represents the angle between the crack and the transversal line, which is used to further judge whether a unidirectional crack is a transversal crack or a longitudinal crack; *T*_ang_ is a supplement to *T*_flg_. When a unidirectional crack has multiple inflection points, the weight of the network crack is judged to increase; *T*_*s*_ is a supplement to the above four indicators. When there are multiple types of cracks in the image, it is divided into three important levels according to the proportion of pixels, and finally the categories are defined according to the high degree of importance.

#### 2.2.2. Crack Image Classification Based on HFS

After multiple membership evaluations of fracture images *C*_*q*_ and *C*_*q*_*j*__, hesitant fuzzy sets *h*_*q*_ and *h*_*q*_*j*__ are formed. *h*_*q*_ and *h*_*q*_*j*__ are used to calculate the hesitating fuzzy similarity sim(*C*_*q*_, *C*_*q*_*j*__). When the similarity is greater, the probability that they is a category is greater. The crack image correlation classification Algorithm 1 based on the hesitant fuzzy set is as follows:

## 3. Results and Discussion

In this section, we mainly discussed the implementation details of the proposed solution and presented experimental results.

### 3.1. Crack Segmentation Experiment Analysis

#### 3.1.1. Dataset and Data Augmentation

To evaluate the performance of this algorithm and other algorithms more objectively, the public road crack dataset Crack500 [31] is selected to evaluate the algorithm. The Crack500 dataset is composed of 500 pavement crack images with an image resolution of 2000 × 1500 or more. It was obtained on the main campus of Temple University using smart devices. Each image is manually marked by an expert to generate corresponding Ground Truth data (GT).

The Crack500 dataset has 250 images for the training set, 50 images for the validation set, and 200 images for the test set. In order to avoid overfitting in the training process, the data need to be augmented. The training set is randomly increased to 2500 images by rotating at 90°, 180°, or 240°. Because of the different sizes of the images, random cropping is used to crop the original image into a size of 256 × 256 pixels.

#### 3.1.2. Training Strategy

The experiment in this article is implemented under the Windows operating system. The deep learning framework is PyTorch, the processor is I5-8500 NVIDIA, and the graphics card is GTX 1660ti. In the experiment, Adam is used to optimise the convergence process, the initial learning rate is 0.0001, the batch size is 12, and the epoch is 50. The learning rate strategy uses an exponential decay method to solve the problem with slow convergence in the network's pretraining through collaborative optimisation of optimisation algorithms and dynamic learning rates.

#### 3.1.3. Data Preprocessing

Due to the low contrast between the cracks in the original image and the surrounding pixels, and the susceptibility to uneven illumination, there is a lot of noise in the image. If the segmentation is performed directly, the discrimination of the same feature will be low, and the existing noise will affect the subsequent segmentation effect. Zhu et al. [32] proposed a defogging algorithm based on image fusion. The underexposed image is obtained on the basis of gamma correction, and then the weight is refused by analyzing the global and local exposure to improve the performance and robustness of image dehazing; Zheng et al. [33] proposed an image defogging algorithm based on adaptive structure decomposition and multiexposure image fusion. On the basis of gamma correction, images with different exposure levels were subjected to adaptive structure decomposition. This algorithm effectively eliminates the noise caused by haze on the image. Inspired by the above, in order to improve the contrast between the crack and the surrounding pixels, improve the uneven illumination, and reduce the image noise, the following preprocessing is performed: (1) grayscale conversion; (2) image standardization; (3) gamma correction, as shown in Figure 7.

#### 3.1.4. Performance Evaluation Index

To better evaluate the performance of the proposed algorithm, this paper uses four indicators of Accuracy, Precision, Dice, and IoU to objectively evaluate the effect of pavement crack segmentation. The calculation formula of the evaluation index is

(12) $$\begin{array}{c} \text{Accuracy}=\frac{\text{TP}+\text{TN}}{\text{TP}+\text{TN}+\text{FP}+\text{FN}},\\ \text{Precision}=\frac{\text{TP}}{\text{TP}+\text{FP}},\\ \text{Dice}=\frac{2\times \text{Precision}\times \text{Recall}}{\text{Precision}+\text{Recall}},\\ \text{IoU}=\frac{\text{Precision}\cap \text{GT}}{\text{Precision}\cup \text{GT}}, \end{array}$$

where true positive examples (TP) and true negative examples (TN) indicate correctly classified cracks and noncrack pixels, respectively; false-positive examples (FP) and false-negative examples (FN) indicate incorrectly classified cracks and noncrack pixels, respectively; GT is a marked image pixel; Accuracy reflects the performance of the algorithm for correctly dividing cracked and noncracked pixels; and Precision represents the performance of the algorithm for correctly dividing the cracked pixels. Dice denotes the harmonic mean of the Precision and Recall.

#### 3.1.5. Loss Function

Since the ratio of cracked pixels to noncracked pixels is highly imbalanced, the effect of cracked areas on the loss is relatively small, resulting in low splitting accuracy of cracked pixels. In order to make the network balance this problem, the focus loss function [34] is introduced, focusing on the crack area and difficult-to-separate samples.

(13) $$\begin{array}{c} \text{focal loss}\left(p_{t}\right)=-\alpha {\left(1-p_{t}\right)}^{\gamma }\log\;p_{t}, \end{array}$$

where *α* is used to balance the imbalance of positive and negative samples between cracks and background areas. If there are few samples of the crack category, the weight of its loss increases. *γ* reduces the influence of easy-to-classify samples on the network model and pays attention to the training of difficult samples to further improve the segmentation accuracy.

Table 1 shows the effect of weight changes on the results on the Crack500 data set. Since *α* and *γ* have a mutual influence, when selecting their values, when the value of *γ* increases, the value of *α* is correspondingly reduced. It can be seen from the experimental results that when the value of *γ* is 1, with the increase of *α*, the four indicators have different degrees of growth. When the value of *γ* is 2, the effect is optimal as *α* increases to 0.25. The above table is the best part of the experimental results. With comprehensive analysis of the values of multiple indicators, the final value of *γ* is 2, and the value of *α* is 0.25.

#### 3.1.6. Result Analysis

*(1) Ablation Experiment*. To verify the effectiveness of the modules in the proposed method, Table 1 shows the effects of different modules on the segmentation results. The following modules are added to verify the effectiveness of the modules based on the U-shaped network with the ResNeXt encoder. The training parameters of each network containing different modules are consistent with the proposed network.

EDA: the high-efficiency dual attention module is added. As seen in Table 1, Precision, Dice, and IoU have increased by 0.47%, 0.12%, and 0.51%, respectively. Therefore, we can conclude that the attention module is effective for pavement crack detection tasks.

MFF: the multiscale feature fusion module is added. As seen in Table 1, Precision, Dice, and IoU have increased by 2.25%, 1.11%, and 1.23%, respectively, which proves the effectiveness of adding the multiscale feature module.

Focal loss: after replacing the cross-entropy loss function with the focal loss function, the experimental results show that Precision, Dice, and IoU increase by 1.66%, 0.87%, and 0.60%, respectively.

The results of the ablation experiment are shown in Table 2. The focus loss function and the multiscale feature fusion module improve the network performance most substantially. The high-efficiency dual attention module contributes to the improvement of Precision and IoU. Due to the small and complex topological structure of the pavement cracks, the focus loss function improves the segmentation quality of the small cracks. The multiscale feature fusion module obtains multiscale context information to solve the complex topological structure presented by the crack image. The high-efficiency dual attention mechanism suppresses noise information, such as shadows and scratches through the importance of the channel and space features, effectively enhancing the characteristic ability of the network.

*(2) Compared with Existing Algorithms*. Qualitative analysis: To verify the performance of MACSNet in road crack detection, the algorithm in this paper is compared with other algorithms on the public dataset Crack500, including U-Net [35], CE-Net [21], DeepLabv3 [24], and DeepLabv3+ [36]. Their data enhancement and training methods use the methods described in 3.1 and 3.2. Figures 8(a)–8(g) show some of the output results.

The segmentation results of each algorithm can be seen directly in Figure 8. When the crack topology in the image is simple, the above five algorithms can segment the cracks well, as shown in the first row of the above figure. When there are shadows, scratches, and other noises in the background of the image, as in the second and third rows, U-Net, DeepLabv3, DeepLabv3+, and CE-Net all have different degrees of crack segmentation discontinuity problems, and MACSNet can segment continuous cracks. The reason may be considering the global context information. When the topological structure of the crack in the image is complex, such as in Lines 4–6, the missed detections of U-Net, DeepLabv3, and CE-Net are more serious. Although DeepLabv3+ missed a few cracks, as seen in the fifth line, it lacks the integrity of the cracks. Contours and MACSNet also add a local importance attention mechanism, which can accurately segment small cracks, extract feature information more abundantly, and qualitatively analyze the effectiveness of MACSNet.

Quantitative analysis: According to the evaluation indicators in Section 3.1.4, the test results are obtained on the public dataset Crack500, as shown in Table 3. Accuracy and Precision alone are not enough to judge the performance of each algorithm for splitting cracks. At the same time, comprehensive evaluation indices Dice and IoU are used to evaluate the performance of each algorithm. It can be seen from Table 2 that MACSNet's Dice is 2.10%, 3.58%, 2.17%, and 1.25% higher than U-Net, CE-Net, DeepLabv3, and DeepLabv3+, respectively. IoU is higher than U-Net, CE-Net, and DeepLabv3, respectively. And DeepLabv3+ is 2.34%, 3.97%, 2.22%, and 1.13% higher. Therefore, it is verified that the effect of MACSNet is substantial, which is consistent with the results of the qualitative analysis.

The time complexity of the MACSNet algorithm proposed in this paper is shown in Table 3. Frames Per Second (FPS) represents how many frames of images the algorithm can process in one second, and we use FPS to represent the time complexity. Although our method is slower than the general segmentation methods U-Net and CE-Net, it is faster than the advanced segmentation method DeepLabv3+. To analyze the reason, we have made a compromise in time complexity in order to improve the segmentation accuracy of the algorithm, but our method can still reach the real-time standard and has obvious advantages in time complexity.

*(3) Compared with Other Advanced Algorithms*. To further illustrate the effectiveness of MACSNet, MACSNet is compared with other advanced methods under the same dataset, and the results are shown in Table 4. In this paper, the MACSNet algorithm's Accuracy, Precision, and IoU values are better than other road crack segmentation algorithms.

### 3.2. Crack Classification Experiment Analysis

#### 3.2.1. Dataset Introduction

In order to verify the effectiveness of the crack classification method based on the hesitant fuzzy set, the dataset in this section selects 948 images from the dataset in Section 3.1. It is divided into four categories: 404 transversal cracks; 276 longitudinal cracks; 57 block cracks; 40 alligator cracks.

#### 3.2.2. Evaluation Index

In order to analyze the effectiveness of the multiattribute fuzzy classification method on crack images, the Recall (R) and Precision (P) are selected to evaluate the image classification results.

**Definition 9 .**

Recall (R) indicates the percentage of the number of images FS that are similar to the input image in the classification results and the number of all similar images in the dataset AS.

(14) $$\begin{array}{c} R=\frac{\text{FS}}{\text{AS}}*100\%. \end{array}$$

**Definition 10 .**

Precision (P), which represents the percentage of the number of images FS that are similar to the input image in the classification results to the number of images NS in the total classification results.

(15) $$\begin{array}{c} P=\frac{\text{FS}}{\text{NS}}*100\%. \end{array}$$

#### 3.2.3. Result Analysis

*(1) Classification Result Analysis*. Definitions 9 and 10 prove that FS represents the number of images retrieved when the similarity to the image to be retrieved is higher than the threshold T. AS represents the number of all similar images in the dataset, and NS represents the total number of retrieved images. For example, there are 276 longitudinal cracks in the 1124 dataset, and the corresponding P and R values are calculated according to the Precision and Recall calculation rules.

It can be concluded from Table 5 that, under different thresholds, the Precision and Recall of the method in this paper are maintained at approximately 84% and 80%, respectively. With the decrease of the threshold, the number of images similar to the input image in the search result and the number of all search result images are increasing, but the former increases more slowly than the latter, which leads to a decrease in the *P*-value and an increase in the R-value. After the analysis, when the threshold is lowered, the massive cracks may be classified as longitudinal cracks, which causes the *P*-value of the algorithm in this paper to decrease.

To further verify the effectiveness of the algorithm in this paper, the difference between the Recall and the Precision of the four categories is obtained through the experiments. When there are different types of cracks in a picture, a larger proportion of the cracks prevail. The experimental results are shown in Table 6.

Judging from the crack classification results in Table 6, the classification algorithm proposed in this paper can basically realize the classification of four types of cracks. The Precision rates of transverse cracks and longitudinal cracks reached 83.85% and 84.09%, respectively, and block and alligator cracks reached 77.98% and 78.38%, respectively. After the analysis, the massive and cracked cracks are affected by the complex geometric structure, as well as the threshold of the average distance between the particles. This paper proposes a crack type classification algorithm based on hesitant fuzzy sets, which can handle the situation where there are multiple crack targets in an image.

*(2) Compared with Other Advanced Algorithms*. In this section, the method in this paper is compared with existing methods using the Crack500 data set. Safaei et al. [37] proposed a tile-based cracking method, applying local threshold technology to each tile. According to the spatial distribution characteristics of crack pixels, the tiles containing cracks are detected, and after fitting a curve, classify longitudinal and transverse cracks by setting the slope threshold, hereinafter referred to as method 1; Song et al. [30] proposed a crack classification method based on a characterization algorithm. Through the connected area labeling algorithm and the spatial distribution of the cracks, the cracks are divided into four types: transversal, longitudinal, block, and alligator. This method effectively detects the crack information in a complex environment, hereinafter referred to as method 2.

The classification results of this research method and other methods are shown in Table 7. The P and R values of method 1 are similar to the method in this paper, but unfortunately, due to the imperfect algorithm, it is impossible to distinguish between massive cracks and cracked cracks. Compared with method 2, the method in this paper only has a slightly lower R-value for transverse fractures, and other indicators are higher than those of method 2. A closer look will reveal that the difference between method 2 and the text method in *P*-value is less than 1%–3%, but the R-value is less than 1%. Analyze the reason: our method adds hesitation on the basis of the connected domain labeling algorithm. Fuzzy feature attributes have a large increase in Precision to a certain extent, but at this time, some fuzzy categories may be introduced to cause a low increase in Recall. The above experimental results show that the method in this paper has a better classification effect than the existing methods.

The time complexity of the hesitant fuzzy set classification algorithm proposed in this paper is shown in Table 6. It can be seen from the table that our method is better than method 1 and is slightly lower than method 2. To analyze the reason, we introduced the hesitant fuzzy attribute on the basis of the connected domain labeling algorithm, which increased the calculation degree of the algorithm and caused our time complexity to be slightly lower than that of method 2. But our method has a better balance between accuracy and time complexity and has obvious advantages compared to methods 1 and 2.

## 4. Conclusion

In the current crack detection methods, most of them only segment the crack images and do not involve classification, but the type of cracks is very important to the evaluation of the road health status, so we propose multiscale attention and HFS crack detection and classification method. This method distributes the weights of the two dimensions of channel and space through cross-channel attention and local importance pooling, so that the network automatically pays more attention to the characteristic information of the crack area and further improves the detection accuracy of the crack. A multiscale feature fusion module is designed to fuse multiscale context information, and the rectangular pooling method is used instead of average pooling to retain important fracture information. This detection method is more suitable for the detection of crack images with unbalanced aspect ratios than existing methods. On this basis, a road crack image classification method based on HFS is designed. On the basis of the connected domain algorithm, using the advantages of HFS in multiattribute decision-making, the membership degree of the cracks is calculated, and the similarity of the cracks is obtained for classification judgement. This classification method uses fuzzy multiattribute special features to further improve classification accuracy. Through comparative experiments, the effectiveness of the above methods is verified. Experimental results show that this method has good crack detection and classification effects, and it has a certain auxiliary effect on the evaluation of road health.

The follow-up work is mainly carried out from the following two aspects: The network training time cost is considered and the lightweight semantic segmentation network is introduced into the multiscale attention segmentation network to achieve faster and accurate binary images. According to the complex topology of the cracks, it is necessary to improve the attribute index and optimise the classification method of crack images, especially for classifying massive cracks and cracked cracks.

## Figures and Tables

**Figure 1:** MACSNet framework.

**Figure 2:** Efficient dual attention module.

**Figure 3:** Multiscale feature fusion module.

**Figure 4:** Decoder module.

**Figure 5:** Fracture image analysis.

**Figure 6:** Centroid angle.

**Figure 7:** Original image and preprocessed image.

**Figure 8:** Segmentation results of each algorithm on the Crack500 dataset. (a) Image. (b) GT. (c) MACSNet. (d) U-Net. (e) DeepLabv3. (f) DeepLabv3+. (g) CE-Net.

**Algorithm 1:** 

**Table 1:** The effect of weight value changes on the results.

*γ*	*α*	Accuracy	Precision	Dice	IoU
-	—	97.12	69.81	65.20	54.12
1	0.70	96.21	70.43	63.75	52.69
1	0.75	96.90	70.49	64.12	53.24
1	0.80	97.12	72.06	66.18	53.73
1	0.85	97.33	73.89	66.93	54.56
1	0.90	97.29	73.60	66.87	54.51
2	0.10	98.35	71.85	65.50	53.22
2	0.15	98.48	**74.30**	66.24	53.90
2	0.20	98.57	74.27	66.91	55.23
2	0.25	**98.62**	74.26	**67.43**	**55.56**
2	0.30	98.61	74.09	67.38	55.51

Bold values are the best performing values.

**Table 2:** Test results of each algorithm's segmentation index on the Crack500 dataset.

EDA	MFF	Focal loss	Precision %	Dice %	IoU %
✓			70.35	65.45	53.73
✓	✓		72.60	66.56	54.96
✓		✓	73.01	66.90	54.89
		✓	71.43	65.36	53.82
	✓	✓	73.86	67.21	55.01
✓	✓	✓	74.26	67.43	55.56

**Table 3:** Test results of each algorithm's segmentation index on the Crack500 dataset.

Algorithm	Accuracy%	Precision%	Dice%	IoU%	FPS
U-Net [35]	96.12	69.88	65.33	53.22	47.49
CE-Net [21]	96.89	70.47	63.85	51.59	43.90
DeepLabv3 [24]	96.91	70.41	65.26	53.34	23.12
DeepLabv3+ [36]	96.94	71.06	66.18	54.43	23.80
MACSNet (our)	98.62	74.26	67.43	55.56	30.91

**Table 4:** Comparison with other advanced methods on the Crack500 dataset.

Algorithm	Accuracy %	Precision %	IoU %
Chen et al. [9]	—	—	51.40
Augustauskas et al. [10]	98.32	64.47	53.34
Cao et al. [8]	N.A	68.05	54.92
MACSNet (our)	98.62	74.26	55.56

**Table 5:** Experimental results under different thresholds.

T (%)	FS	NS	AS	P (%)	R (%)
90	215	251	276	85.66	77.90
85	218	259	276	84.17	78.99
80	222	264	276	84.09	80.43
75	225	269	276	83.64	81.52

**Table 6:** Experimental results of fracture classification based on hesitant fuzzy sets.

Crack category	FS	NS	AS	P (%)	R (%)
T	322	384	404	83.85	79.70
V	222	264	276	84.09	80.43
M	170	218	228	77.98	74.56
C	29	37	40	78.38	72.50
Mean				81.08	76.80

**Table 7:** Performance comparison with the other two methods.

Category	T		V		M		C		FPS
	P%	R%	P%	R%	P%	R%	P%	R%	
Method 1	83.40	80.02	83.40	80.02	—	—	—	—	0.50
Method 2	82.91	**80.77**	83.94	79.96	75.61	74.23	74.95	72.19	2.13
Our	**83.85**	79.70	**84.09**	**80.43**	**77.98**	**74.56**	**78.38**	**72.50**	2.04

## Data Availability

The data that support the findings of this study are available upon request.
